This article has been retracted.

# A Retrospective Cohort Study of the Efficacy, Safety, and Clinical Value of 6-TG versus 6-MP Maintenance Therapy in Children with Acute Lymphoblastic Leukemia

**DOI:** 10.1155/2022/7580642

**Published:** 2022-08-21

**Authors:** Minghui Tu, Aiming Zhang, Li Hu, Feng Wang

**Affiliations:** Department of Pediatrics, Xiangyang No. 1 People's Hospital, Hubei University of Medicine, Xiangyang 441000, China

## Abstract

**Objective:**

To explore the efficacy, safety, and clinical value of 6-TG versus 6-MP when treating childhood acute lymphoblastic leukemia (ALL).

**Methods:**

The study period was from January 2017 to June 2021. The subjects of this study were 100 children with ALL who were treated in our hospital. According to different intervention methods, the children who received 6-MP maintenance therapy were selected as the control group, with a total of 57 cases. Children with TG maintenance therapy were included in the research group, a total of 43 cases. The ICNS recurrence rate, non-ICNS recurrence rate, first remission mortality rate, secondary malignant tumor, and other indicators were compared.

**Results:**

First of all, we compared the effective rate: complete remission (CR), partial remission, and nonremission in the study group, and the effective rate was 87.5%. In the control group, there were CR, partial remission, and no remission, and the effective rate was 65.5%. The effective rate of the study group was higher, and the difference between groups was statistically significant (*P* < 0.05). There were 55 cases of failure in the study group, with an incidence of 21.91%. There were 42 cases of total failure events in the control group, the incidence rate was 18.02%, and there exhibited no remarkable difference (*P* > 0.05). In the study group, 6 cases died in the first remission, with a fatality rate of 2.39%, while there exhibited no death in the control group. The mortality in the first remission period in the study group was lower (*P* < 0.05). The overall recurrence rate of the study group was 5.57%, while that of the control group was 11.15%. The overall recurrence rate of the study group was lower, and the difference between groups was statistically significant (*P* < 0.05). The recurrence rate of ICNS was 2.14% in the study group and 2.98% in the control group, and there exhibited no remarkable difference (*P* > 0.05). The non-ICNS recurrence rate was 3.43% in the study group and 7.17% in the control group. There exhibited no remarkable difference (*P* > 0.05). The incidence of secondary malignant tumor events was 0.85% in the study group and 1.59% in the control group. There exhibited no remarkable difference (*P* > 0.05). The incidence of hepatic vein occlusive disease was 7.29% in the study group and 2.39% in the control group. The incidence of hepatic vein occlusive disease in the study group was higher, and the difference between groups was statistically significant (*P* < 0.05). Finally, we compared the incidence of adverse reactions. In the study group, there were 12 cases of oral mucosal damage, 7 cases of liver function damage, 6 cases of infection, 10 cases of myelosuppression, 9 cases of gastrointestinal reaction, and 4 cases of skin damage; the incidence rate was 23.17%. In the control group, there were 12 cases of oral mucosal damage, 7 cases of liver function damage, 6 cases of infection, 10 cases of myelosuppression, 9 cases of gastrointestinal reaction, and 4 cases of skin damage, with an incidence of 19.12%. There exhibited no remarkable difference in the incidence of adverse reactions (*P* > 0.05).

**Conclusion:**

6-TG maintenance therapy in children with ALL can enhance the overall effective rate, can reduce the first remission mortality and the total recurrence rate, and will not increase the overall incidence of adverse reactions, but the incidence of reversible or irreversible hepatic veno-occlusive disease is remarkably increased, which has a certain clinical value.

**Background:**

Treatment-related hepatotoxicity and myelosuppression remain formidable challenges for clinicians. Pharmacokinetic studies found that 6-TG has a more direct intracellular activation pathway, shorter cytotoxic time, and stronger potency than 6-MP. Therefore, this study investigated the efficacy, safety, and clinical value of 6-TG and 6-MP in the treatment of children with ALL.

## 1. Introduction

Acute lymphoblastic leukemia (ALL) is one of the most common malignant hematological tumors [1]. In recent years, its incidence is increasing, especially in children. The annual incidence of childhood ALL in China is about 0.67/100000. ALL is one of the main causes of death in children. With the continuous improvement and optimization of clinical treatment, the prognosis of ALL has been remarkably enhanced, but 15% to 20% of children and about 50% of adult patients will have drug-resistant recurrence after induction of chemotherapeutic drugs [2]. Once recurrence occurs, the cure rate will be less than 40%. Drug-resistant recurrence has always been the primary factor leading to treatment failure and high mortality in children with ALL. The problem of recurrence has increasingly become a hot topic in the research of childhood ALL. At present, the most important treatment of ALL is the use of chemotherapeutic drugs to induce remission and consolidation treatment [3]. ALL-induced remission phase is the use of high-dose chemotherapy drugs combined therapy; after this stage, most patients will get CR and then through low-dose thiopurine long-term maintenance to consolidate treatment. Thiopurine drugs have been widely adopted when treating leukemia since they were put on the market in the 1950s and achieved good clinical results; thiopurine drugs are nucleotide-like drugs, which need to be transformed into bioactive nucleotide-like products mercapto-guanine nucleotides (thioguanine nucleotides (6-TGNs)) by metabolic enzymes in vivo to exert their efficacy [4]. They mainly act in the S phase of tumor cells, can be inserted into chromosome replication, and can inhibit cellular purine metabolism, so as to kill tumor cells. Usually, thiopurine drugs are used for consolidation therapy for about 2-2.5 years. During this treatment, if some key metabolic enzymes or genes in the drug metabolic pathway are mutated and result in functional changes, then leukemia cells will be resistant to the treatment of thiopurine drugs, and tumor cells will soon relapse. Thiopurine drugs mainly include two kinds of drugs: one is 6-MT and its derivative azathioprine (AZA), and the other is 6-TG. All three are widely adopted when treating leukemia and autoimmune diseases, but because the toxicity of 6-TG is higher compared to of 6-MP and AZA, 6-TG is generally only adopted in patients with failed or intolerant treatment of 6-MP and AZA. Thiopurine drugs are prodrugs, and their metabolism in vivo is a complex process [5]. AZA can be rapidly converted to 6-mercaptopurine under the action of glutathione S-transferase. 6-Thioguanine nucleotides and 6-thioguanosine nucleoside monophosphate are produced by hypoxanthine guanine phosphate ribosyltransferase and 6-thioguanine nucleoside monophosphate, respectively. 6-Thio-hypoxanthine nucleotides are converted to 6-thio-xanthine nucleotides under the catalysis of hypoxanthine nucleotide dehydrogenase and to 6-thioguanosine nucleoside monophosphate under the catalysis of guanine nucleotide synthetase, which can be phosphorylated to form diphosphate and triphosphate called 6-TGNs [6]. Thiopurine drugs can be catalyzed by mercaptopurine methyltransferase, xanthine oxidase (XO), and cytoplasmic 5-nucleotidase-II to form inactive components, all of which can reduce the drug effect. 6-MP has been adopted in the clinical treatment of ALL in children for more than 60 years, but its mechanism has not been fully elucidated [7].

Hepatotoxicity and myelosuppression related to treatment are still great challenges for clinicians. Due to the lack of direct parameters to monitor the efficacy of patients, so the intensity of treatment is difficult to grasp, clinicians still need to further adjust the treatment plan in order to reduce mercaptopurine drug resistance [8]. Since 1980, pharmacokinetic studies have found that 6-TG has a more direct intracellular activation pathway, shorter cytotoxic time, and stronger potency than 6-MP, which theoretically explains why 6-TG may be more effective [9]. Since 1990, there have been clinical studies to compare the efficacy of the two drugs. Some animal experimental data also preliminarily suggest that 6-TG may be more effective than 6-MP. This study retrospectively analyzed the efficacy, safety, and clinical value of 6-TG versus 6-MP when treating childhood ALL [10].

## 2. Patients and Methods

### 2.1. Normal Information

The study period was from January 2017 to June 2021. The subjects of this study were 100 children with ALL who were treated in our hospital. According to different intervention methods, the children who received 6-MP maintenance therapy were selected as the control group, with a total of 57 cases, and 43 children who received maintenance therapy with 6-TG were included in the study group. In the control group, the age ranged from 1 to 18 years old, with an average of 11.42 ± 2.18 years, including 33 males and 24 females. In the study group, the age ranged from 1 to 18 years old, with an average of 11.57 ± 2.04 years, including 25 males and 18 females. There exhibited no remarkable difference in general data. This study was permitted by the Medical Ethics Association of our hospital, and all patients noticed informed consent.

Inclusion criteria: (1) diagnosed as ALL, (2) less than 18 years old, (3) no previous history of cognitive impairment and mental illness, and (4) informed consent.

Exclusion criteria: (1) patients ≥ 18 years old, (2) received antileukemia treatment before treatment, (3) secondary ALL, (4) complicated with other neoplastic diseases and genetic metabolic diseases, (5) patients with previous history of mental illness and cognitive impairment or suspected cognitive impairment, and (6) patients with severe hepatorenal dysfunction, severe infection, and severe diabetes.

### 2.2. Treatment Methods

The control group received maintenance therapy with 6-MP: standard regimen VDLP and vincristine (VCR) 1.5 mg/m^2^ were used in the induced remission phase, once a week × 4 times; daunorubicin (DNR) 30 mg/m^2^, once a week, 2~3 times in total; asparaginase (L-ASP) 6000–10000 U/m^2^ once every other day, 6–8 times in total; prednisone was administered orally at 60 mg/m^2^ three times a day for a total of 28 days with a 7-day reduction in stopping time. During the consolidation phase, CAT regimen was adopted, cyclophosphamide (CTX) 800–1000/m^2^. On the first day, cytarabine (Ara-C) 100 mg/m^2^/day × 7 days twice a day (every 12 hours), subcutaneous injection, thioguanine (6-TG), or thiopurine (6-MP) 75 mg/m^2^/day and oral administration in the evening × 7 days. The maintenance treatment phase consisted of 6-MP+MTX/VD+sheathing regimen, intramuscular injection of methotrexate (MTX) at 20–30 mg/m^2^ per week for 3 weeks, and oral administration of thiopurine (6-MP) at 75 mg/m^2^ per day for 21 days; vincristine (VCR) 1.5 mg/m^2^ dosing followed by prednisone 45 mg/m^2^ daily for 7 days. In this way, the cycle was repeated once every 4 weeks, and the doses of methotrexate (MTX) and 6-MP were adjusted according to the white blood cell counts in the peripheral blood of individuals to maintain the white blood cell counts at (2.8–3.0) × 10^9^/L. The total course of chemotherapy ranges from two to two and a half years. In the study group, 6-TG was used for maintenance therapy: the treatment plan in the induced remission phase and consolidation phase was completely the same as that in the control group, and the maintenance therapy phase was treated with 6 murine TGG plus MTX+intrathecal injection of methotrexate (MTX) intramuscular injection of 20~30 mg/m^2^ once a week for 3 weeks, while 6-TG was taken orally for 21 days every day for 40 mg/m^2^; vincristine (VCR) 1.5 mg/m^2^ dosing followed by prednisone 45 mg/m^2^ daily for 7 days. In this way, the cycle was repeated every 4 weeks, and the doses of methotrexate (MTX) and mercaptopurine (6-MP) were adjusted according to the individual peripheral blood white blood cell count to maintain the white blood cell count at (2.8–3.0) × 10^9^/L.

### 2.3. Observation Index

#### 2.3.1. Treatment Effective Rate

Complete remission (CR): the clinical symptoms basically disappeared; the results of peripheral hemogram (male) Hb ≥ 110 g/L or (female) Hb ≥ 100 g/L > 100 g/L, absolute neutrophils ≥ 1.5 × 10^9^/L, no leukemic cells in peripheral blood. The myelogram results suggest that the original+immature lymphocytes are less than 5%, and the red blood cells and megakaryocytes are normal. Partial remission (PR): myelogram results suggest that primary+immature lymphocytes are less than 5% and 20%. Or one of the clinical symptoms and hemogram was not completely relieved. No remission: the children did not reach partial remission. Total effective rate = (CR + PR) cases/total cases × 100%.

#### 2.3.2. Overall Failure Rate and Fatality Rate in the First Remission Period

Failure events are defined as the occurrence of death, recurrence, or secondary malignant tumor from the beginning of maintenance therapy. Excluding the data of early death and induced remission death, the death case in the remission stage was the fatality rate of the first remission stage.

#### 2.3.3. ICNS Recurrence Rate and Non-ICNS Recurrence Rate

The recurrence rate of isolated central nervous system (ICNS) is defined as the number of WBC in cerebrospinal fluid (CSF) which is 0.005 × 10^9^ (5/*μ*L) or higher. Meanwhile, primordial cells are found on centrifuge smears, and there is no evidence of leukemia in other parts. The recurrence rate of ICNS was defined as recurrence in other sites such as bone marrow and testis, excluding multiple site recurrence.

#### 2.3.4. Incidence of Secondary Malignant Tumor Events and Hepatic Veno-Occlusive Disease

The second malignant tumor events and the incidence of hepatic veno-occlusive disease were counted during the follow-up period.

#### 2.3.5. Incidence of Adverse Reactions

The oral mucosal damage, liver function damage, infection, myelosuppression, gastrointestinal reaction, and skin damage were calculated.

### 2.4. Statistical Analysis

The data were analyzed by SPSS 21.0 statistical software, and the measurement data were presented by ($\bar{x}\pm s$). The *t*-test of independent samples was adopted for the comparison. Paired *t*-test was adopted for the comparison before and after treatment. The counting data were presented by example *n* (%). *P* < 0.05 indicated that the difference between groups was statistically significant.

## 3. Results

### 3.1. Overall Efficiency

Firstly, we compared the effective rate: CR, partial remission and nonremission in the study group, and the effective rate was 87.5%. The effective rate of CR, partial remission and nonremission in the control group was 65.5%, the effective rate in the study group was higher, and the difference between groups was statistically significant (*P* < 0.05). All the data results are indicated in Figure 1.

### 3.2. Comparison of Overall Failure Rate and Fatality Rate in the First Remission Period

There were 55 cases of failure in the study group, with an incidence of 21.91%. There were 42 cases of total failure events in the control group, with an incidence of 18.02%. There exhibited no remarkable difference in data (*P* > 0.05). In the study group, 6 cases died in the first remission, with a fatality rate of 2.39%. There exhibited no death in the control group in the first remission period, and the mortality in the study group was lower, and the difference between groups was statistically significant (*P* < 0.05). All the data results are indicated in Table 1.

### 3.3. Comparison of Overall Recurrence Rate, ICNS Recurrence Rate, and Non-ICNS Recurrence Rate

The overall recurrence rate of the study group was 5.57%; the overall recurrence rate of the control group was 11.15%. Compared between groups, the overall recurrence rate of the study group was lower, and the difference between groups was statistically significant (*P* < 0.05). The recurrence rate of ICNS in the study group and the control group was 2.14% and 2.98%, respectively. There exhibited no statistically remarkable difference (*P* > 0.05). The non-ICNS recurrence rate was 3.43% in the study group and 7.17% in the control group. There exhibited no remarkable difference (*P* > 0.05). All the data results are indicated in Table 2.

### 3.4. Incidence of Secondary Malignant Tumor Events and Hepatic Veno-Occlusive Disease

The incidence of secondary malignant tumor events in the study group was 0.85%, while that in the control group was 1.59%. There exhibited no remarkable difference in data (*P* > 0.05). The incidence of hepatic vein occlusive disease was 7.29% in the study group and 2.39% in the control group, the incidence of hepatic vein occlusive disease in the study group was higher, and the difference between groups was statistically significant (*P* < 0.05). All the data results are indicated in Table 3.

### 3.5. Comparison of Adverse Reactions

Finally, we compared the incidence of adverse reactions. In the study group, there were 12 cases of oral mucosal damage, 7 cases of liver function damage, 6 cases of infection, 10 cases of myelosuppression, 9 cases of gastrointestinal reaction, and 4 cases of skin damage; the incidence rate was 23.17%. In the control group, there were 12 cases of oral mucosal damage, 7 cases of liver function damage, 6 cases of infection, 10 cases of myelosuppression, 9 cases of gastrointestinal reaction, and 4 cases of skin damage, with an incidence of 19.12%. There exhibited no remarkable difference in the incidence of adverse reactions (*P* > 0.05). All the data results are indicated in Figure 2.

## 4. Discussion

Leukemia is a malignant proliferative disease of the hematopoietic system, which is characterized by the stagnation of hematopoietic cells in the primitive low differentiation stage and malignant clonal proliferation, and the proliferated leukemic cells do not have normal function [11]. The pathogenic mechanism of leukemia cells is that these abnormal cells enter the blood circulation and destroy normal blood cells in various tissues and organs of the body. The above conditions will induce the body's immune cells and immune organs to react, resulting in varying degrees of liver and spleen lymphadenopathy and bone pain and other clinical manifestations, which can lead to anemia, hemorrhage, infection, etc. [12]. At present, the etiology and pathogenesis of leukemia are not fully understood, which may be related to virus infection, physical and chemical factors stimulation, and genetic defects. In China, leukemia is the most common malignant tumor in children. According to the survey, there are about 15000 new leukemia children in China every year, of which 70% to 80% are ALL [13]. It is gratifying to note that over the past half a century, with the continuous development of immunology, molecular biology, and genetic technology, human beings have gained a deeper understanding of the etiology and pathogenesis of leukemia. With the progress of diagnosis and treatment technology and the continuous improvement of treatment, through multidrug and multicourse combined chemotherapy, the success rate of treatment of childhood leukemia has increased year by year [14]. The total cure rate of ALL in children is close to 80%. Therefore, the current goal of the treatment of ALL in children is no longer simply to achieve short-term remission, but to strive to achieve long-term disease-free survival and enhance the quality of life in the future. This not only depends on the accurate clinical risk classification and the choice of chemotherapy intensity but also requires continuous summary and analysis from previous diagnosis and treatment, accumulating more treatment experience, and closely combining laboratory research with clinical research [15]. Research and experience will be combined and organically applied to future treatment.

Induced remission therapy is the first course of ALL chemotherapy [16]. Killing leukemic cells to the maximum extent in a short period of time and achieving CR as soon as possible are the key to long-term event-free survival (EFS). Different induction treatment options choose different drugs, generally for the combination of 4 or 7 drugs, namely, daunorubicin, vincristine, asparaginase, and glucocorticoid [17]. Meanwhile, because of the high tumor load in the initial treatment, a series of side effects caused by the destruction and dissolution of tumor cells, and the side effects of chemotherapeutic drugs, there is a high risk of treatment. Therefore, the choice of chemotherapy should not only pay attention to the intensity of treatment but also reduce the toxic and side effects caused by chemotherapy as much as possible and avoid the related death and the occurrence of secondary tumor caused by chemotherapy, that is, on the premise of ensuring the effect of treatment, enhance the quality of life of children as far as possible, in order to achieve individual treatment as the goal [18].

Mercaptopurine drugs show classic antimetabolic cytotoxicity and increase cell lethality by prolonging the action time of the drugs [19]. 6-MP and 6-TG are two inactive prodrugs, which need to activate cytotoxic metabolites to exert their efficacy in the process of metabolism. The process of purine metabolism is complex, and the mercaptan methylation pathway competes with the nucleotide metabolite synthesis pathway, which mainly includes three competitive pathways: oxidation pathway, methyl pathway, and nucleotide metabolite formation pathway [20]. Nucleotide metabolites are catalyzed by hypoxanthine guanine phosphate ribose transferase (HGPRT) and mercaptopurine methyltransferase (TPMT). The oxidation of mercaptopurine is catalyzed by XO, as indicated in Figure 1. The activity of XO enzyme in the liver is very high, but it is lacking in blood cells. 6-MP is first metabolized by liver XO enzyme and finally transformed into two main intracellular toxic metabolites, including thioguanine nucleotides (TGN) and methylmercaptopurine metabolites [21]. TGN then infiltrates into DNA or RNA to exert antitumor effect. Methylated mercaptopurine metabolites are mainly synthesized by TPMT enzyme, including meTIMP and meTGMP. The former is a potent inhibitor of purine de novo synthesis (DNPS), which makes 6-MP have remarkable toxicity. However, 6-TG does not inhibit the DNPS pathway, so the latter has little effect on its metabolism, and the toxicity of 6-TG mainly depends on the infiltration of TGN into DNA at a higher concentration [22]. Preclinical drug toxicity studies indicated that the cytotoxicity threshold of 6-MP was about 1 *μ*mol/L, and the maximum cytotoxicity concentration was 10 *μ*mol/L. The threshold of 6-TG was 0.05 *μ*mol/L, the maximum cytotoxic concentration was 0.5 *μ*mol/L, and its IC50 was 15 times lower compared to 6-MP. 6-TG is not the direct substrate of XO. 6-TG can directly activate the intracellular TGN pathway, and one of the important activation pathways is the process of thiomethylation by TPMT [23]. Therefore, 6-TG has more remarkable cytotoxicity than 6-MP. In addition, 6-TG can kill cells more quickly, and its minimum drug exposure time is much less compared to of 6-MP. In metabolism, 6-TG and 6-MP both form thioxanthine (TX), which is the first metabolite produced in the production of thiuric acid [24]. 6-MP is converted into 6-TX by XO, while 6-TG is converted into 6-TX by guanosinase. In order to reduce the oral dose of 6-MP during treatment, patients often need to take XO inhibitors, but 6-TG does not [25]. Adamson et al. believe that 6-TG may have stronger efficacy, but it needs to be confirmed by a large number of prospective clinical randomized controlled trials. In 1996, Lennard et al. proposed that erythrocyte TGN concentration is independent of other prognostic variables of ALL, including age, immunophenotype of leukemia, white blood cell count at diagnosis, test scheme, and sex [26]. Plasma half-life and S-phase-dependent pharmacokinetics indicate that the bioactive concentration and exposure time of TGN are very important for tumor cell killing, and monitoring this metabolite has important clinical significance [27]. A large number of clinical randomized controlled trials confirmed that the erythrocyte TGN accumulation concentration in the 6-TG group was remarkably higher compared to that in the 6-MP group, but there exhibited no difference in 3TGN concentration range of systematic evaluation of the efficacy and safety of leukocyte 6-thioguanine when treating childhood ALL [28]. Although white blood cells are closer to target lymphocytes than red blood cells, conventional chemotherapy drugs lead to myelosuppression in children, and the monitoring of leukocyte metabolites is not feasible [29]. The metabolism of drugs in red blood cells and white blood cells is different. Mature red blood cells have no purine synthesis pathway, mainly through an efficient remedial mechanism to metabolize purine precursors [30]. Meanwhile, the life cycle of red blood cells is longer compared to of white blood cells, so drug metabolites accumulate and cycle throughout the whole life cycle of red blood cells. TGN is the active product of intrahepatic metabolism and extrahepatic purine metabolism (erythrocytes), which directly reflects the difference between the metabolism of two mercaptopurine drugs and the remedial ability of erythrocytes [31]. There is no evidence that the level of leukocyte TGN in children with ALL taking 6-MP is lower compared to in children taking 6-TG. Other studies suggest that the cytotoxic effect of 6-MP is not entirely based on the formation of TGN, and the concentration of TGN may simply reflect the ability of erythrocytes to directly metabolize 6-TG to TGN [32]. When the dose of 6-MP increased, the metabolic mode changed from TGN to methylated (TIN), and its dose intensity should also be an important factor affecting drug metabolism [33]. In order to explore the effect of 6-MP dose intensity on 6-MP drug metabolism, Bell et al. included 226 children who were treated with 6-MP in 2004 [34]. Among them, 110 children were given daily dose of 75 mg/m^2^, and the control group was treated with fractionated dose 37.5 mg/m^2^. The results indicated that the mean erythrocyte methylated thiopurine metabolite level of 6-MP in the daily dose group was higher compared to the divided dose group [35]. The relationship between methylated mercaptopurine metabolites and TGN will serve as a mature part of elucidating the clinical outcome of 6-MP. In clinic, the treatment of mercaptopurine in children with ALL is complicated in terms of dosage, course of treatment, drug selection, and remediation of side effects [36]. The therapeutic effect of ALL was also related to disease grade, sex, and age of patients. According to the risk grade of children, intrathecal injection of chemotherapeutic drugs was given to prophylaxis treatment of central nervous system (ICNS) leukemia. At present, there is no evidence that 6-TG is better than 6-MP in improving quality of life, prolonging survival time, and reducing mortality in children with ALL. This study provides some important clues for maintaining the drug selection of mercaptopurine drugs during the treatment period. There is no definite clinical effect of using 6-TG instead of 6-MP when treating ALL in children during maintenance therapy, and further research is needed to provide evidence-based basis for the clinical treatment of 6-TG [37]. Therefore, it is suggested that when using 6-TG, the monitoring of blood active metabolites and side effects should be strengthened. Anti-infection, liver protection, reduction of jaundice, and use of low molecular weight heparin can enhance the prognosis of children. If anemia is serious, red blood cell transfusion can be given according to the general condition and laboratory examination. When severe thrombocytopenia occurs, single platelet suspension should be given, and 6-TG treatment should be stopped in time [38]. High-dose and long-term use of 6-TG will lead to chronic hepatotoxicity and portal hypertension in children with ALL. It was originally described in the randomized controlled trial (MRCALL97) studied by Vora et al. in 2006 [39]. 11% of the children in the 6-TG group developed nonfatal HVOD. There is no systematic study on the mechanism of liver injury induced by thiopurine. The main clinical manifestations of HVOD induced by 6-TG are mild hepatomegaly, hyperbilirubinemia, elevated transaminase, thrombocytopenia, and portal hypertension, which are common in hematological and solid tumor chemotherapy and hematopoietic stem cell transplantation pretreatment, which can endanger children's life in severe cases. The vast majority of children (>90%) indicated transient mild hepatomegaly, mild to moderate hyperbilirubinemia with elevated transaminase, and moderate to severe thrombocytopenia [40]. One child initially indicated the clinical characteristics of hepatic venule occlusive disease, and the autopsy biopsy confirmed that he died of adenovirus infection, so it is necessary to pay attention to the differentiation of the two diseases. Portal hypertension is mainly due to liver tissue fibrosis or nodular regeneration and proliferation around the portal vein caused by injury of hepatic sinusoidal endothelial cells, which eventually leads to hepatic sinusoidal outflow tract obstruction [41]. Clinically, most patients with hepatic sinusoidal obstruction syndrome have to stop using 6-TG after a few years of treatment because of remarkable HSOS, which is a common complication of autologous and allogeneic hematopoietic stem cell transplantation (HSCT). It is also seen in patients with nephroblastoma and rhabdomyosarcoma undergoing chemotherapy. However, HSOS is rare in routine chemotherapy for other malignant tumors in children [42]. Doppler ultrasound is also helpful for the diagnosis of HSOS, including hepatomegaly, splenomegaly, ascites, thickening of gallbladder wall, elevated resistance index of hepatic artery, and blood reflux signal in portal vein. In recent years, the clinical use of multislice spiral CT combined with MPR and liver CTA imaging is helpful to the differential diagnosis and clinical evaluation of HSOS [43]. Most of the reversible HVOD patients in the American CCG-1952 test have only HSOS manifestations and do not have mature clinical manifestations of HVOD or meet the pathological diagnostic criteria [44]. 6-TG-related HSOS that occurred during Baixiaoan treatment was associated with glutathione depletion and oxidative stress in hepatocytes. Other chemotherapeutic drugs including the interaction of vincristine and the increased concentration of homocysteine induced by methotrexate may reduce anticoagulant protein levels [45]. Myelosuppression is the most recent toxic reaction of mercaptopurine drugs. Recent studies have indicated that leukopenia, neutropenia, thrombocytopenia, and elevated transaminase are all remarkably correlated with the dose of mercaptopurine drugs. The same idea can be found in the study put forward by Chen et al. [46]. They have applied new methods in the study, and the conclusions drawn can also give some support to this study. There are some limitations in this study. First, the sample size of this study is not large and it is a single-center study, so bias is inevitable. In future research, we will carry out multicenter, large-sample prospective studies, or more valuable conclusions can be drawn.

In summary, 6-TG maintenance therapy in children with ALL can enhance the overall effective rate, can reduce the first remission mortality and the total recurrence rate, and will not increase the overall incidence of adverse reactions, but the incidence of reversible or irreversible hepatic venous occlusive disease is remarkably increased, which has a certain clinical application value.

## Figures and Tables

**Figure 1:** Comparison of overall efficiency between two groups.

**Figure 2:** Comparison of adverse reactions between two groups.

**Table 1:** Comparison of overall failure event rate and mortality in the first remission period [*n*(%)].

Grouping	*N*	Overall failure event rate	Mortality in the first remission period
Control group	251	55 (21.91)	6 (2.39)
Research group	233	42 (18.02)	0 (0)
*t*		1.139	3.856
*P*		>0.05	<0.05

**Table 2:** Comparison of overall recurrence rate, ICNS recurrence rate, and non-ICNS recurrence rate [*n*(%)].

Grouping	*N*	ICNS relapse rate	Non-ICNS relapse rate	Overall recurrence rate
Control group	251	10 (3.98)	18 (7.17)	28 (11.15)
Research group	233	5 (2.14)	8 (3.43)	13 (5.57)
*t*		1.359	3.321	4.845
*P*		0.243	0.068	0.027

**Table 3:** Comparison of the incidence of secondary malignant tumor events and hepatic veno-occlusive disease [*n*(%)].

Grouping	*N*	Incidence of secondary malignant tumor events	Incidence of hepatic vein occlusive disease
Control group	251	4 (1.59)	6 (2.39)
Research group	233	2 (0.85)	17 (7.29)
*t*		0.533	6.424
*P*		0.465	0.011

## Data Availability

The datasets used and analyzed during the current study are available from the corresponding author upon reasonable request.
